The article "Impact of Closed Operation Strategies on Profit of Core Enterprise in Closed Supply Chain for Vegetables: A System Dynamics Approach" was published in 2022. Journal: Comput Intell Neurosci.

# Impact of Closed Operation Strategies on Profit of Core Enterprise in Closed Supply Chain for Vegetables: A System Dynamics Approach

**DOI:** 10.1155/2022/2721176

**Published:** 2022-05-20

**Authors:** Lingling Liu, Vatcharapol Sukhotu

**Affiliations:** School of Management, Asian Institute of Technology, Pathumthani, Thailand

## Abstract

This paper aims to, from the new perspective of the impact of closed operation strategies on profit of core enterprise, adopt the theory of closed supply chain, find solutions to maximize control of vegetable quality and safety, and improve profit of core enterprises in the supply chain. Two of the most representative vegetables exported from Yunnan Province to Thailand are selected for this empirical study. And the system dynamics model witnesses the completion of simulation and forecast under eight schemes, respectively. Through contrastive analysis, the development trends of the two vegetables come to the same conclusion; that is, simultaneously strengthening the three closed strategies enables the creation of the biggest economic benefit for core enterprises in vegetable supply chain from Yunnan Province to Thailand.

## 1. Introduction

### 1.1. Background

Nowadays, the safety incidents of agricultural products occur frequently in many countries, and how to effectively control the quality and safety of them has become the common concern all over the world. The quality and safety of vegetables are closely related to the operation level of the supply chain management, which is becoming the whole process management of the supply chain from “farm-to-table” [1]. Therefore, exploring an innovative operations mode for vegetable supply chain has paved the way for solving the problems of vegetable quality and safety. In 2006, Chinese scholars first proposed “Closed Supply Chain,” an exclusive form of supply chain that has developed to an advanced stage, which shared a new thinking with us to solve the problems of vegetable quality and safety from the perspective of supply chain process management. The reason why it is “closed” indicates that the existing supply chain is mostly “open” to anyone who wants to purse vegetable business, and there is no high-standard threshold for enterprises entering the supply chain, and no explicit stipulation for the quality and safety of vegetable products [2].

Thailand and China are the major participates of economic cooperation in Greater Mekong Subregion (GMS) and China-ASEAN Free Trade Area (CAFTA); the agricultural product structures of two countries are complementary. China is Thailand's second largest export market and the largest source of imports [3]. Yunnan Province is located in southwest boarder of China and is a pivotal gateway from Thailand to China. In Thailand, the vegetable acreage accounts for 0.735% of all the land area [4], and the vegetable cultivation is mainly concentrated in the northern provinces of Chiang Mai and Chiang Rai with 20 varieties such as basil, fennel, capsicum, balsam pea, crispy eggplant, long eggplant, yellow-fruit nightshade, and parsley. Compared with the steady supply of vegetables all year round in Yunnan Province, the rainy season greatly reduces vegetable production in Thailand from May to November every year; vegetables import from Yunnan Province has therefore become a rigid demand of Thai markets. Specifically, Thailand has been steadily importing over 20 varieties of vegetables from Yunnan Province, including *Capsicum frutescens*, potato, tomato, pea, celery, broccoli, onion, Chinese chives, cabbage, and lettuce. According to the data of Kunming Customs [5], the volumes and values of Yunnan's vegetables exported to Thailand from 2015 to 2020 showed a steady upward trend (see Table 1).

The article "Impact of Closed Operation Strategies on Profit of Core Enterprise in Closed Supply Chain for Vegetables: A System Dynamics Approach" was published in 2022. Journal: Comput Intell Neurosci.

According to statistics of Kunming Customs, the total amount of vegetables exported from Yunnan Province to Thailand in 2020 was 241,045 tons, of which *Capsicum frutescens* 29,648.5 tons (12.3%) and broccoli was 27,720.2 tons (11.5%), as shown in Figure 1. Meanwhile, the total export value of Yunnan vegetables exported to Thailand in 2020 reached 192 million dollars, of which *Capsicum frutescens* was 19.78 million dollars (10.3%) and broccoli was 21.12 million dollars (11.0%), as shown in Figure 2. The export volume and export value of the two vegetables ranked the top two in 2020. Although without an absolute advantage, they accounted for a high proportion, which could be representative to a certain extent. From the field survey, we know that *Capsicum frutescens* and broccoli have come to the two most representative vegetables in this supply chain, because they fit the favor of taste for Thai people and have a great demand in Thai markets.

After the completion of Kunming-Bangkok Road in December 2013, coupled with a series of port facilitation measures, it takes an average of 24 hours for Yunnan vegetables to be transported from the production base to the entry port, Chiang Khong in Thailand, and then 36 hours to be delivered to the supermarket shelves or wholesale markets in Thailand, which is 1.5 times shorter than that in the past, and the loss rate of goods has also dropped from 35% to 2% [3].

### 1.2. Problem Definition and Motivation

With the continuous expansion of vegetable trade between Yunnan Province and Thailand, we are increasingly aware of the severe challenges brought by the traditional operations mode of supply chain. The risks of quality and safety of Yunnan vegetables frequently occur in planting, processing and distribution; even some of products cannot reach the import standards of Thailand. In second half of 2020, the sampling inspection results from Yunnan Administration for Market Regulation show that in 74,989 vegetable samples, the quantity of unqualified is 3,353, a defect rate of 4.5%, and the total economic losses absorbed by growers and processing enterprises reached 0.201 million dollars [6]. Since the outbreak of COVID-19, Thai Customs execute the clearance procedures for Yunnan vegetables more strictly, and each batch of vegetables imported from China must be inspected. The quality and safety of vegetables from Yunnan has always been a bottleneck that baffles vegetable enterprises, as well as the profits of the whole supply chain. However, the traditional operations of vegetable supply chain in Yunnan Province fail to meet the market's requirements for quality and safety of vegetables.

The article "Impact of Closed Operation Strategies on Profit of Core Enterprise in Closed Supply Chain for Vegetables: A System Dynamics Approach" was published in 2022. Journal: Comput Intell Neurosci.

Therefore, aiming to strictly control the quality and safety of vegetables, as well as to improve the profit of member enterprises in vegetable supply chain, plenty of studies have proposed to implement some strategies for quality control in the whole process of vegetable supply chain, which mainly refer to three dimensions: certificate of market access, multistage quality inspection, and information traceability system [1, 2, 7–10]. In addition, the profit, as we know, is a primary indicator to measure the enterprise competence. However, there have been no studies on profit of core enterprises in vegetable supply chain, and how to apply the closed strategies to maximize the profit of core enterprises in vegetable supply chain is unknown. Thus, adopting the theory of closed supply chain and analyzing the impact of closed strategies on profit are expected to benefit core enterprises to translate demand into profits to large potentials, in order to maximally control the quality and safety of vegetables, and enhance the competitiveness of vegetable supply chain from Yunnan Province to Thailand.

For this concern, based on the above puzzles in either practice or theory, in order to work out solutions to this bottleneck, this study attempts to use SD to simulate and forecast the impact of closed strategies on profit of core enterprises in closed supply chain for vegetables. Taking vegetable trade from Yunnan Province to Thailand as a case, a comprehensive SD model is constructed by Vensim software. Based on the constructed platform, we predicted the future trend of profits in off-season of a year (180 days). Then, the model is used to simulate and forecast the profits under eight schemes.

The article "Impact of Closed Operation Strategies on Profit of Core Enterprise in Closed Supply Chain for Vegetables: A System Dynamics Approach" was published in 2022. Journal: Comput Intell Neurosci.

### 1.3. Contribution and Content Organization

This study holds the potential to provide a unified SD-based research framework which can systematically and comprehensively analyze the impacts of closed strategies and future trends in vegetable supply chain. In terms of case application, this study proposes a model for core enterprises in vegetable supply chain to calculate and predict long-term profits. By establishing causality and flow diagram to simulate the impacts of three closed strategies on core enterprises, it provides policy implications for managing and controlling the quality and safety of agricultural products. Furthermore, this is an adaptable platform which can be applied to different categories of agricultural products supply chain and can be adjusted according to the needs of decision makers.

This study is organized as follows.  Section 2 reviews and analyzes the literature regarding the related theories.  Section 3 sets up system dynamics model, and Section 4 makes simulation and forecasting. The paper is concluded by conclusion and recommendation in Section 5.

## 2. Literature Review

This section presents the current research in closed supply chain and closed operation strategies and quality and safety control for vegetable supply chain, as well as core enterprises.

### 2.1. Closed Supply Chain and Closed Operation Strategies

#### 2.1.1. Closed Supply Chain

This concept was first proposed by the scholar of Nankai University in China in 2006, who argues that the closed supply chain enables to implement access control for node enterprises on the basis of strategic cooperation of supply chain and to establish unified operation standards in terms of supply chain business process which can be effectively monitored and tracked in real time. The quality information traceability can be realized in this form of supply chain. As an innovative operational system, starting from the market demand of agricultural products, the closed supply chain is oriented by product quality and safety, and follows the circulation characteristics and market system characteristics of agricultural products to entirely guarantee the quality and safety of agricultural products [2].

In European and American researches, the terms of “quality and safety control” or “quality management” are widely used in supply chain management which refer that the strict entry and management systems are implemented among the supply chain members including Good Agricultural Practices (GAP), Technical Standard Order (TSO), Real Time Monitoring and dynamic tracing prediction, and traceability supply chain system [11]. By using these techniques, the relatively stable strategic alliance relationships and standardized operational procedures are established among supply chain members [1,12]. Meanwhile, the closed supply chain is considered as the superior form of the traditional supply chain. Compared to the traditional one, it highly focuses on food quality and safety control through each node of the supply chain whose value lies in supplement and innovation [2]. The existing supply chain management represents a key principle to improve cost, time, and service level [13]. However, the closed supply chain emphasizes vertically expanding uniform standards of quality and safety among upstream and downstream of the supply chain [1]. Such expansion provides efficient designs that form multiple dimensions of quality control system from food sources, government regulation, management model, and information system [10].

The article "Impact of Closed Operation Strategies on Profit of Core Enterprise in Closed Supply Chain for Vegetables: A System Dynamics Approach" was published in 2022. Journal: Comput Intell Neurosci.

According to the connotation of closed supply chain, the closed supply chain does not refer to a market closure but emphasizes a higher threshold to enter the supply chain, as well as a higher level of supply chain cooperation and collaboration [1]. The differences between closed supply chain and other four types of supply chain are illustrated in Table 2. It can be seen that, besides the obvious orientation of food quality and safety, the closed supply chain has higher operation cost and average capacity of flexible production compared with the other four types of supply chain and needs a strong supervision from the third party; however, it displays better stability [14,15].

#### 2.1.2. Closed Operation Strategies of Vegetable Supply Chain

The closed operation strategies of vegetable supply chain in this study consist of three aspects, referring to the certificate of market access, multistage quality inspection, and information traceability system, which enable them to be simultaneously operated in a framework and constitute the operation mode of closed supply chain [1, 9].

  Strategy 1: certificate of market access:
  The certificate of market access is a management system in vegetable supply chain, whose purpose is to restrict the circulation of vegetables that fail to meet the quality and safety standards, and to maximally control the quality and safety of vegetables. Specifically, only producers that meet the prescribed conditions are allowed to engage in production and business activities, and only agricultural products that meet the prescribed conditions are allowed to be produced and distributed in the supply chain [7, 8, 16]. Currently, the market access system of agricultural products in most countries follows three ways: one is based on the receipts, invoices, or tickets before entering the market; the second is based on on-site quality testing; the third one is based on various forms of quality and safety certificates. All of the three types of market access are oriented by quality testing [15].
  Strategy 2: multistage quality inspection:
  The multistage quality inspection is a quality inspection system that combines the proactive quality control of core enterprises (processing and export enterprises) with the compulsory quality control of government, and involves the whole process testing of vegetable supply chain [1]. Furthermore, according to unified quality testing standards, the multistage quality inspection system is established by core enterprises in each stage of vegetable supply chain to prevent problem products from entering the retail terminal [17]. The government quality supervision department, on the other hand, conducts mandatory testing and regulation to vegetable products, and more often, the multistage quality inspection system is jointly built by both government and member enterprises [7, 18].
  Strategy 3: information traceability system:
  The information traceability system is a quality information traceability platform which is mainly invested by government, with the model of platform e-commerce. It makes mandatory entry for members of closed supply chain, where each member enterprise is enabled to timely query and share the demands, production, and price information of the main vegetable varieties [1, 2, 8, 10, 19].

The article "Impact of Closed Operation Strategies on Profit of Core Enterprise in Closed Supply Chain for Vegetables: A System Dynamics Approach" was published in 2022. Journal: Comput Intell Neurosci.

### 2.2. Quality and Safety Control for Vegetable Supply Chain

The vegetable supply chain is regarded as a network structure in which vegetables are distributed from farmers, processing enterprises, distribution centers, wholesalers, and retailers to customers. As one of subcategories of agricultural products, with their particular natural attributes, vegetables promote the reintegration of the original supply chain and improve the efficiency and value of the supply chain [17]. Vegetable industry is recognized as a typical labor-intensive industry. As a result of short freshness, higher moisture content, being perishable, and being affected by natural conditions, vegetables have come to depend on pesticides and fertilizers, and agricultural film and hormones are also put into the production process, which has greatly affected the quality and safety of vegetables [20]. Information asymmetry between producers and consumers may lead to waste or inefficiency in vegetable supply chain. Therefore, the accurate and real-time information is the key factor to ensure the efficiency and balance of vegetable supply chain [21]. It is worth noting that focus of this subject mainly lies in two aspects, namely, circulation model and cost control, as well as logistics network and traceability system.

The article "Impact of Closed Operation Strategies on Profit of Core Enterprise in Closed Supply Chain for Vegetables: A System Dynamics Approach" was published in 2022. Journal: Comput Intell Neurosci.

Considering the quality and safety control for vegetable supply chain which is a complex and dynamic issue, many scholars are committed to the modeling and analysis of circulation model and cost control. Zhang [15] builds a circulation pattern for vegetables in Tianjin based on closed supply chain management, which refers to the fact that based on supply chain management technologies, a network has been managed consisting of farmers, cooperatives, core enterprises, distributors and sales enterprises, logistics companies, and processing and circulation enterprises, by involving consciousness of quality and safety, environmental protection, and green management throughout the whole process of vegetable circulation. Frank et al. [22] analyze the problems faced by the model of “farmers + enterprises” by adopting principal-agent theory and then propose a model of “agricultural association + enterprises” to guarantee the quality and safety of agricultural products as well as the farmers' financial benefits. Yang [23] proposes that there are two basic forms of vegetable supply chain in China, namely, the vegetable supply chain system of direct-to-consumer with farmers market terminal and the vegetable supply chain system with chain supermarket terminal. These two models complement each other; however, each of them has its own disadvantages which are due to the higher price, long distance, and the inconvenient transportation. Liu and Zhang [24] analyze the operation characteristics and cost control of three typical models in closed supply chain of agricultural products, namely, wholesaler-dominated model, manufacturer-dominated model, and government-dominated model. In addition, dynamic programming is used to solve the cost value in different supply chain stages under a fixed cost standard. Then, the time series method is adopted to forecast and renew the future activity costs. Meanwhile, the programming is used to calculate the optimal costs and dynamic cost trend, which offers a new way to analyze the dynamic costs in vegetable closed supply chain. Sun and Zhang [25] conduct a case study of eggplants and investigate the cost structure and profit distribution of four links of eggplant supply chain in China, including procurement, transport, wholesale and retail. Alam and Khatun [26] analyze the effects of COVID-19 pandemic on vegetable industry in Bangladesh. They indicate that the price of yield has dropped by more than the half resulting in huge loss for vegetable growers. The decreased income increases farmers' likelihood of vulnerability and food insecurity and poses a challenge to continued produce. “Cash support” is more important than “food support” in order to keep vegetable farmers in farming, to ensure a ready supply of necessary low-cost resources, and to help fight against the upcoming food shortage. Rakesh et al. [27] propose a unique fuzzy multi-criteria decision making approach for improving the vegetable losses through cold-third party logistics providers (CTPLs) evaluation and selection process. The result shows that “refrigerator and loading capacity” and “knowledge and onformation technology management” are most significant in the selection of CTPLs.

The article "Impact of Closed Operation Strategies on Profit of Core Enterprise in Closed Supply Chain for Vegetables: A System Dynamics Approach" was published in 2022. Journal: Comput Intell Neurosci.

For logistics network and traceability system of this problem, many researchers have improved and optimized the deep learning framework of models and algorithms and then applied them to the daily operation of vegetable supply chain. Qiu [8] constructs optimization models of logistics network for closed supply chain of green agricultural products with deterministic and optional logistics conditions, respectively, from the perspective of vegetable quantity and quality losses. Wang et al. [28] study the distribution plan of large-scale supermarket and specialty vegetables circulation enterprises in vegetable supply chain. Then aiming to minimize logistics costs and carbon emissions, the multi-objective programming model is established and the scheme of solving the model is given. Alfred [29] establishes the data collecting process and the Bayesian model for vegetable safety traceability and alerting system based on the critical control point analysis. In addition, the model facilitates the quality monitoring and forecasting, which serves as a reliable systematic means for vegetable supply “from farm to table.” Gong and Zhang [30] propose a supply chain management system for pollution-free vegetables based on RFID in order to realize the traceability, automation and information management for pollution-free vegetables. Then, they optimize the circulation management process through RFID technologies, so as to improve the safety and management efficiency of pollution-free vegetables. Chandrasekaran and Raghuram [10] analyze the factors that contribute to postharvest losses of the vegetable supply chain by developing an ISM model, especially in an Indian context. Also, they compare the ISM model to the model proposed based on the loading patterns of responses, and provide recommendations on how to improve the real-time tracking to make timely interventions.

### 2.3. Core Enterprises

Due to the asymmetry of information and resources, the competitive advantages of some enterprises become more prominent in greater competition in the market, thus forming the core enterprises, which are in the dominant position in the industrial cluster [31]. With the increasing influence in supply chain, core enterprises have been given attention and studied. The connotation of core enterprise is mainly divided into three perspectives: supply chain, industrial cluster, and innovation network, and this paper only focuses on the first aspect.

The article "Impact of Closed Operation Strategies on Profit of Core Enterprise in Closed Supply Chain for Vegetables: A System Dynamics Approach" was published in 2022. Journal: Comput Intell Neurosci.

From the perspective of supply chain, most of the research aims to analyze the characteristics and functions of core enterprises. For example, Prahalad and Hamel [32] propose that the core enterprise has key technologies or products that are hard to be imitated by competitors in the supply chain, that is, the root for core enterprise to achieve sustainable and healthy growth and finally gain competitive advantages in the field. Harland [33] argues that core enterprise is generally manufacturing or retail enterprise of larger scale and implements related diversification based on its core competence. Bendiner [34] defines the core enterprise as a corporate that has the influence in the operations of supply chain, leads the business dealings with other enterprises, and has inimitable advantages to form the core competitiveness. Ma [35] indicates that. as the central link of the supply chain, the core enterprise possesses key resources and information and plays a leading role in supply chain operations. The core enterprise promotes the formation of strategic cooperative relations in the supply chain by exerting its considerable influence on guiding and controlling the market. Ahuja [31] believes that, as the unique core resource is available for core enterprises, it enables us to control the procedure and rhythm of the supply chain operations, allocate, and integrate resources in the supply chain, so as to promote the overall core competitiveness of the supply chain.

The core enterprise in this study refers to the agricultural enterprise which works in vegetable processing and export, and reaches the prescribed standards in terms of scale, technical force, and financial strength. It enables us to lead the implementation of the closed operations mode of vegetable supply chain [20]. As the leader of the supply chain, the processing and export enterprise connects farmers, importers, and wholesalers. It purchases vegetables from farmers, vegetable cooperative, or its own production base, and then it processes and transports vegetables to the port by outsourcing to the third-party logistics. It also looks for and signs cooperation agreements with demanders and importers of Thailand.

### 2.4. Summary and Research gap

From the review findings above, it can be found that the related theories and methods have been quite extensive on the quality and safety control for vegetable supply chain. As for the contents, the studies mainly focus on methods of quality and safety control for vegetable supply chain, information asymmetry, production and consumption behavior, cost benefit analysis, and quality and safety regulation of vegetable products, as well as characteristic and function of core enterprise, which have acquired abundant and valuable achievements. In addition, for research methods, the current studies concern is to set up theoretical models in order to analysis the construction, evolution, and development of operations mode of closed supply chain. However, research gaps in this field mainly exist in the following aspects. (i) There is a lack of a unified method or research framework that can systematically and comprehensively analyze the profit of core enterprise in vegetable supply chain. (ii) Few studies have involved the specific closed operation strategies, and there is no research on the combination of closed operation strategies with core enterprises. (iii) Any empirical study on impact of closed operation strategies on profit of closed supply chain is still suspended so that serious data in vegetable business cannot be collected with accuracy and timeliness. To fill these gaps, system dynamics (SD) can be an appropriate method. Compared with the existing solutions mentioned above, the SD has the advantage of combining qualitative and quantitative analysis to solve complex system dynamic problems and to better simulate the decision-making process as it is easy to link observable patterns of behavior of a system to microlevel structure [36].

The article "Impact of Closed Operation Strategies on Profit of Core Enterprise in Closed Supply Chain for Vegetables: A System Dynamics Approach" was published in 2022. Journal: Comput Intell Neurosci.

## 3. Methods and Materials

### 3.1. Introduction to System Dynamics and Vensim

System dynamics (SD) founded by Professor J. W. Forrester of Massachusetts Institute of Technology (MIT) in 1956 is a discipline that analyzes information feedback systems. It is an important quantitative approach for evaluating the resources carrying capacity [37]. The model mainly reflects the causal feedback relationship between the variables of each module in a system by establishing the first-order differential equations, simulating the development of different plans and forecasting the decision variables by system dynamics model. Then, these decision variables are served as the index system of carrying capacity, and, by using evaluation methods, the optimal development plan and corresponding state of carrying capacity are obtained in the form of comparing schemes [38].

Vensim is a type of system dynamics software that is developed by Ventana Company and runs under Windows. It mainly has version of Vensim PLE, PLE Plus, Professional DSS, and Model Reader, which is suitable for different users, as well as some applicable functions such as graphical modeling, composite simulation, array variables, validation, sensitivity testing, and model optimization. Compared with other versions, Vensim DSS has more comprehensive configurations, which adds an interface development tool for creating management flight simulators, external functions and macros, compiled simulations, and more [39].

The article "Impact of Closed Operation Strategies on Profit of Core Enterprise in Closed Supply Chain for Vegetables: A System Dynamics Approach" was published in 2022. Journal: Comput Intell Neurosci.

### 3.2. Boundary of Profit System for Core Enterprises

Aiming at simplifying the complexity of the system, a complete system can be decomposed into several subsystems by SD simulation [38]. To study the profit system of core enterprises by SD model, in the first place, the boundary of the system should be clearly defined. Since the vegetable supply chain from Yunnan Province to Thailand is characterized as a long-term, seasonal, and continuous system and the profit system of core enterprises has been affected by many factors, it is difficult to consider all factors when modeling a system's structure, which requires us to remove some factors that have less impact. Thus, this study proposes the following hypotheses for modeling:

(1) The operations of vegetable supply chain are considered as a continuous and gradual process, which is a cycle and closed system. Firstly, the vegetable supply chain in this study refers to an industrial chain composed of production base, processing and export enterprises (core enterprises), import enterprises and wholesalers. Vegetable products gradually flow in each node enterprise, which is a continuous supply process from upstream to downstream of the supply chain. Secondly, the word of “closed” means the supply chain does not open to all enterprises, but it only allows those whose products meet relevant quality and safety standards to be the supply chain members. That is to say, any enterprise failing to meet the relevant quality standards will be not allowed to enter the supply chain, and no product is permitted to be moved to the next link of the supply chain if it fails to meet the relevant quality standards. It emphasizes a higher threshold to enter the supply chain, as well as a higher level of supply chain cooperation and collaboration [1].
(2) Due to the numerous and complex links involved in the vegetable supply chain, this model only focuses on the profit of core enterprises (the processing and export enterprises), and the main research objects involve the core enterprises, import enterprises, and wholesalers, except other nodes and consumers in the supply chain.
(3) As the cross-level ordering of each node in the vegetable supply chain, in order to simplify the operations procedure, the situation that customers directly order vegetable products from farmers through e-platform is not considered in this model.
(4) As Yunnan vegetables are the daily necessities of Thai people, the demand and sales of Yunnan vegetables in Thai markets have been relatively stable in recent years, and there are periodic variations in the off-season and peak season every year. Therefore, this model focuses on the tendency of profit in off-season, in which data in 180 days are collected and the dynamic changes are studied.
(5) Based on the logistics flow of vegetables in major node enterprises, the profit system of core enterprises is divided into four subsystems in this study, including S1: inventory of processing enterprises, S2: qualified inventory in core enterprises, S3: inventory of import enterprises, and S4: inventory of wholesalers. Specific contents are as follows:
    S1: inventory of processing enterprises:
    It refers to the difference between the quantities of vegetables received by processing enterprises from production bases or farmers and the qualified inventory of processing enterprises after quality testing by the core enterprise.
    S2: qualified inventory in core enterprises:
    In S2, the qualified vegetable products from the processing enterprises are transported to the cold storage warehouse of the core enterprise, by which forms the quantities of vegetables received by core enterprises. The qualified inventory in core enterprises refers to the difference between the quantities of vegetables received by core enterprises and the amount of vegetables in transit from Yunnan Province to Thailand.
    S3: inventory of import enterprises:
    In this phase, the vegetables are transported to the warehouses of Thai importers after quality inspections by both Yunnan Customs and Thailand Customs. The inventory of import enterprises refers to the difference between the quantities received by import enterprises and the amount of vegetables in transit from import enterprises to wholesalers.
    S4: inventory of wholesalers:
    It refers to the difference between the amount of vegetables in transit from import enterprises to the three largest wholesalers and the amount of ex-warehouse in wholesalers.

The article "Impact of Closed Operation Strategies on Profit of Core Enterprise in Closed Supply Chain for Vegetables: A System Dynamics Approach" was published in 2022. Journal: Comput Intell Neurosci.

The framework of profit system of core enterprises is shown in Figure 3. What we do next is to conduct a preliminary causal analysis of the relationship between each influencing factor in order to find out the positive and negative feedback in the system.

### 3.3. Influencing Factors and Causal Diagram

#### 3.3.1. S1: Inventory of Processing Enterprises

S1 is mainly affected by 20 factors. The causality diagram is shown in Figure 4, and the 14 main causality paths are described as follows:

1. Accuracy of demand forecasting-Supply side of vegetable production-Unqualified rate of quality inspection I: core enterprises inspection-Reject ratio in production-Unqualified products-Quantities received by processing enterprises-Inventory of processing enterprises-Qualified inventory of processing enterprises
2. Accuracy of demand forecasting-Supply side of vegetable production-Unqualified rate of quality inspection I: core enterprises inspection-Reject ratio in production-Unqualified products-Quantities received by processing enterprises-Percent defective of processing-Unqualified amount of processing-Internal failure costs-Total costs of core enterprises
3. Accuracy of demand forecasting-Supply side of vegetable production-Unqualified rate of quality inspection I: core enterprises inspection-Reject ratio in production-Unqualified products-Quantities received by processing enterprises-Conversion costs-Total costs of core enterprises
4. Accuracy of demand forecasting-Supply side of vegetable production-Unqualified rate of quality inspection I: core enterprises inspection-Reject ratio in production-Unqualified products-Quantities received by processing enterprises-Acquisition costs-Total costs of core enterprises
5. Quality certification system-Qualified rate of quality inspection II: government sampling inspection-Percent defective of processing-Unqualified amount of processing-Costs of quality certification-Total costs of core enterprises
6. Quality certification system-Qualified rate of quality inspection I: core enterprises inspection-Reject ratio in production- Unqualified products-Quantities received by processing enterprises-Inventory of processing enterprises-Qualified inventory of processing enterprises
7. Quality certification system-Qualified rate of quality inspection I: core enterprises inspection-Reject ratio in production-Unqualified products-Quantities received by processing enterprises-Total costs of core enterprises
8. Time for ordering control-Quantities received by processing enterprises-Inventory of processing enterprises-Qualified inventory of processing enterprises
9. Technical innovation-Percent defective of processing-Percent defective of processing-Unqualified amount of processing-Internal failure costs-Total costs of core enterprises
10. Technical innovation-Reject ratio in production-Unqualified products-Quantities received by processing enterprises-Total costs of core enterprises
11. Technical innovation-Reject ratio in production-Unqualified products-Quantities received by processing enterprises-Inventory of processing enterprises-Qualified inventory of processing enterprises
12. Backward integration-Acquisition price-Acquisition costs-Total costs of core enterprises
13. Backward integration-Reject ratio in production-Unqualified products-Quantities received by processing enterprises-Total costs of core enterprises
14. Backward integration-Reject ratio in production-Unqualified products-Quantities received by processing enterprises-Inventory of processing enterprises-Qualified inventory of processing enterprises

The article "Impact of Closed Operation Strategies on Profit of Core Enterprise in Closed Supply Chain for Vegetables: A System Dynamics Approach" was published in 2022. Journal: Comput Intell Neurosci.

#### 3.3.2. S2: Qualified Inventory in Core Enterprises

S2 is mainly affected by 17 factors. The causality diagram is shown in Figure 5, and the 8 main causality paths are described as follows:

1. Product information traceability system-Quality certification system-Qualified rate of quality inspection I: core enterprises inspection-Costs of quality certification-Total costs of core enterprises-Profits
2. Product information traceability system-Quality certification system-Qualified rate of quality inspection I: core enterprises inspection-Test costs of core enterprises-Total costs of core enterprises-Profits
3. Product information traceability system-Costs of product information traceability system-Total costs of core enterprises-Profits
4. Qualified inventory in core enterprises-Inventory costs-Total costs of core enterprises-Profits
5. Qualified inventory in core enterprises-Amount of vegetables in transit I-Export taxes & fees-Total costs of core enterprises-Profits
6. Amount of vegetables in transit I-Total revenues of export-Profits
7. Transport convenience-Transport time-Damage rate of goods-Amount of damage in transmit for core enterprises-Transport costs-Total costs of core enterprises-Profits
8. Cold chain logistics technologies-Damage rate of goods-Amount of damage in transmit for core enterprises-Transport costs-Total costs of core enterprises-Profits

#### 3.3.3. S3: Inventory of Import Enterprises

S3 is mainly affected by 10 factors. The causality diagram is shown in Figure 6, and the 7 main causality paths are described as follows:

1. Qualified rate of quality inspection III: Yunnan Customs inspection-Costs of quality certification-Total costs of core enterprises-Profits
2. Qualified rate of quality inspection IV: Thai Customs inspection-Costs of quality certification-Total costs of core enterprises-Profits
3. Qualified rate of quality inspection III: Yunnan Customs inspection-Quantities received by import enterprises-Inventory of import enterprises-Amount of vegetables in transit II
4. Qualified rate of quality inspection IV: Thai Customs inspection-Quantities received by import enterprises-Inventory of import enterprises-Amount of vegetables in transit II
5. Inventory of import enterprises-Costs of product information traceability system-Total costs of core enterprises-Profits
6. Transport time-Damage rate of goods-Transport costs-Total costs of core enterprises-Profits
7. Cold chain logistics technologies-Damage rate of goods-Transport costs-Total costs of core enterprises-Profits

The article "Impact of Closed Operation Strategies on Profit of Core Enterprise in Closed Supply Chain for Vegetables: A System Dynamics Approach" was published in 2022. Journal: Comput Intell Neurosci.

#### 3.3.4. S4: Inventory of Wholesalers

S4 is mainly affected by 11 factors. The causality diagram is shown in Figure 7, and the 5 main causality paths are described as follows:

1. Quantities demanded of primary wholesalers-Market forecasting for vegetable sales-Costs of product information traceability system-Total costs of core enterprises-Profits
2. Quantities demanded of primary wholesalers-Market forecasting for vegetable sales-Amount of vegetables in transit II-Damage rate of goods- Inventory of wholesalers-Amount of ex-warehouse in wholesalers-Quantities received by retailers
3. Transport time-Damage rate of goods-Transport costs-Total costs of core enterprises-Profits
4. Cold chain logistics technologies-Damage rate of goods-Transport costs-Total costs of core enterprises-Profits
5. Qualified rate of quality inspection V: sampling inspection in Thai markets-Costs of quality certification-Total costs of core enterprises-Profits

By integrating the above four subsystems, this study attempts to construct a causal relationship diagram of the profit system for core enterprises in vegetable supply chain from Yunnan Province to Thailand, which is shown in Figure 8.

### 3.4. Parameters, Equations and Flow Diagram

#### 3.4.1. Parameters Setting

By using Vensim DSS Version 6.4E, 95 indicators, including level variables, auxiliary variables, and constants, are selected and a system dynamics model is established for determining the impact of closed strategies on profit of core enterprises in the closed supply chain for vegetables. Although vegetable prices vary every day according to the quantity ordered, the demand and sales of Yunnan vegetables in Thai markets have been relatively stable in recent years, as mentioned previously, there are periodic variations in the off-season and peak season every year. Therefore, this model focuses on profit in the off-season, in which the time span is set to 180 days, the initial time is 0, the final time is 180, and the unit for time is 1 day.

The observation time of data in the model lasts from the middle of November to the middle of May in both 2019 and 2020, and the main sources are from Yunnan statistical yearbook, Yunnan Administration for Market Regulation, China Monthly Exports and Imports, Kunming Custom, National Statistical Office Thailand, Thai Customs, and Ministry of Commerce Thailand. Meanwhile, some of the existing research achievements are referred to as relevant parameters in this model. Since the model involves a lot of historical data which need to be sorted out and calculated, the constant parameters are determined by arithmetic averaging of statistical data, as shown below:

1. Export price = 1280 $US/ton
2. Basic transport time = 1.5 day
3. Processing time = 0.4 day
4. Qualified inspection rate, unit inventory cost = 9.7 $US/ton
5. Unit conversion cost = 31.79 $US/ton
6. Inspection time of export enterprises = 0.1 day
7. Costs of quality certification I: production base = 2.87 $US/day
8. Costs of quality certification II: processing enterprises = 5.52 $US/day
9. Unit added-value tax to enter Thailand = 15.88 $US/ton
10. Qualified rate of quality inspection III: Yunnan Customs inspection = 0.98
11. Qualified rate of quality inspection IV: Thai Customs inspection = 0.98
12. Total vegetable imported = 1380 ton/day
13. Transport time to markets = 0.9 day
14. Qualified rate of quality inspection V: sampling inspection in Thai markets = 0.97

In addition, some auxiliary variables are given based on the calculation method in actual operation and expert consultation, and the function relationships of some important variables in the model are mainly expressed by the IF THEN ELSE function, INTEG function, SMOOTH function, and DELAY1 function. The flow diagram of this system is shown in Figure 9, and the main equations are shown below.

The article "Impact of Closed Operation Strategies on Profit of Core Enterprise in Closed Supply Chain for Vegetables: A System Dynamics Approach" was published in 2022. Journal: Comput Intell Neurosci.

#### 3.4.2. Structure of Inventory

In the field of engineering technology, many problems can be transformed into the first kind Fredholm integral equation in [40]

(1) $$\begin{array}{c} \int_{b}^{a}k\left(x,t\right)g\left(t\right)dt=f\left(x\right), \end{array}$$

where *k*(*x*, *t*) and *f*(*x*) are known functions, *a* and *b* denote upper and lower bound constant of integration, and *k*(*x*, *t*) is usually called the kernel function of the integral equation, which determines the basic properties of the integral equation. *f*(*x*) is called the free term of the integral equation and *g*(*x*) is the function to be solved.

With the further developments of fractional order differential equations in the applied sciences, the space fractional order diffusion equations can be used to solve a number of multimodal function optimization; for example, Lee and Prenter [41] solve the numerical solution of the first kind of Fredholm integral equation by means of finite rank and replacing *T*_*x*_=*y* with *T*_*n*_*X*=*y*_*n*_ , *n*=1,2,… (*T*, *T*_*n*_ can be regarded as an operator from *L*_2_[*a*, *b*] to *L*_2_[*c*, *d*] or from *L*_*∞*_[*a*, *b*] to *L*_*∞*_[*c*, *d*]). Maleknejad and Saeedipoor [42] proposed a numerical direct method based on hybrid Block-Pulse functions and Legendre polynomials to solve the first kind of Fredholm integral equation. In addition, Zhang and Yuan [43] estimated the equation parameters by using the Niche Ant Colony Algorithm (NACA) based on fitness sharing principle and verify its efficiency.

The article "Impact of Closed Operation Strategies on Profit of Core Enterprise in Closed Supply Chain for Vegetables: A System Dynamics Approach" was published in 2022. Journal: Comput Intell Neurosci.

In system dynamics models, inventory variables accumulate or integrate their flow variables; the net flow into the inventory is the rate of change for the inventory variable. This structure is represented in (2) as an integral equation.

(2) $$\begin{array}{c} Inventory=\int_{t_{0}}^{t_{1}}\left(Inflows-outflows\right)dt+Invenroty\left(t_{0}\right), \end{array}$$

where Inflows represent the value of the inflow at any time *t* between the initial time *t*_0_ and the current time *t*_1_.

#### 3.4.3. Structure of Profit Rate

The mathematical formulations related to the profit rate and prices are provided as follows. The related notation list is shown in Table 3.

(3) $$\begin{array}{c} P_{i}\left(t\right)=\int_{t_{0}}^{t_{1}}\left[CP_{i}\left(t\right)\right]dt+P_{i}\left(0\right)\;i=1,2, \end{array}$$

(4) $$\begin{array}{c} P_{1}\left(t\right)=\max\left\{0,C\left(1+PR_{1}\left(t\right)\right)\right\}, \end{array}$$

(5) $$\begin{array}{c} P_{2}\left(t\right)=\max\left\{0,P_{1}\left(1+PR_{2}\left(t\right)\right)\right\}. \end{array}$$

Profit rate of the main supply chain member is defined as an inventory variable named *P*_*i*_(*t*) according to (3). Price values in export and wholesaler market are formulated as non-negative auxiliary variables in (4) and (5), respectively.

Based on literature research and field survey, the mathematical formulations pertaining to effects of supply/demand balance on profit rate are provided as follows. The basic modeling logic is based on Sterman's model for a single market [44].

(6) $$\begin{array}{c} CP_{i}\left(t\right)=De\;lay\left[IP_{i}\left(t\right),d\right]-PR_{i}\left(t\right)\;i=1,2, \end{array}$$

(7) $$\begin{array}{c} IP_{i}\left(t\right)=PR_{i}\left(t\right)\cdot EB_{i}\left(t\right)\;i=1,2, \end{array}$$

(8) $$\begin{array}{c} EB_{i}\left(t\right)={\left[B_{i}\left(t\right)\right]}^{Si}\;i=1,2, \end{array}$$

(9) $$\begin{array}{c} B_{1}\left(t\right)=\frac{DS\left(t\right)}{S\left(t\right)+Import}, \end{array}$$

(10) $$\begin{array}{c} B_{2}\left(t\right)=\frac{D\left(t\right)}{min\left\{DS\left(t\right),S\left(t\right)\right\}}. \end{array}$$

By (5), if there is a discrepancy between the desired (*IP*_*i*_(*t*)) and actual state of profit rate (*PR*_*i*_(*t*)), corrective action is initiated to bring the state of the profit rate variable back in line with the desired value according to (7).

The article "Impact of Closed Operation Strategies on Profit of Core Enterprise in Closed Supply Chain for Vegetables: A System Dynamics Approach" was published in 2022. Journal: Comput Intell Neurosci.

For better representation of the reality in this supply chain, this paper considers the inflation and its effect on price values. As information transfer is often delayed in each node of supply chain, the effect of demand/supply balance on price is considered with a delay of 1 day. The delay parameters are approximate values obtained based on information provided by expert consultation.

The effective term of demand/supply balance (*EB*_*i*_(*t*)) appearing in (7) is defined in (8). By (9) and (10), demand/supply balance terms are defined as the related demand divided by the whole supply in the related market. By (9), *B*_1_(*t*) is calculated by dividing *DS*(*t*) by the total supply of core enterprise, which is the summation of *S*(*t*) and Import.

In modeling of *B*_2_(*t*), as shown in (9), the retailers' demand (*D*(*t*)) is divided by the actual supply, which is the minimum of demand and supply in the export market.

#### 3.4.4. Function Formulas in Each Subsystem

1. Market forecasting for vegetable sales = SMOOTH (Sales volume of vegetables, Time for quick response)
2. Qualified rate of quality inspection I: core enterprises inspection = IF THEN ELSE (0.971 *∗* Quality certification system ≥ 1, 1, 0.971 *∗* Quality certification system)
3. Quantities received by processing enterprises = SMOOTH (Supply side of vegetable production-Unqualified products, Time for ordering control)
4. Time for ordering control = 1 *∗* (1 − Product information traceability system) Qualified rate of quality inspection I: core enterprises inspection = IF THEN ELSE (0.971 *∗* Quality certification system ≥ 1, 1, 0.971 *∗* Quality certification system)
5. Test costs of processing enterprises = IF THEN ELSE (Qualified rate of quality inspection I: core enterprises inspection >0, 12.03, 0)
6. Qualified rate of quality inspection II: government sampling inspection = IF THEN ELSE (0.905 *∗* Sampling inspection of agricultural sectors *∗* Quality certification system ≥ 1, 1, 0.905 *∗* Sampling inspection of agricultural sectors *∗* Quality certification system)
7. Qualified inventory of processing enterprises = DELAY1 (Inventory of processing enterprises-Unqualified amount of processing, Inspection time of export enterprises + Processing time)
8. Costs of quality certification = IF THEN ELSE (Quality certification system > 0, Costs of quality certification I: production base + Costs of quality certification II: processing enterprises, 0)
9. Rate of cost change = IF THEN ELSE (Total costs of core enterprises = 0, 0, (Total costs of core enterprises-DELAY1 (Total costs of core enterprises, 1))/Total costs of core enterprises)
10. Amount of ex-warehouse in processing enterprises = IF THEN ELSE (Qualified inventory in core enterprises ≥ 800, Qualified inventory in core enterprises, 0)
11. Rate of change in receiving government subsidies = IF THEN ELSE (Government subsidies = 0, 0, (Government subsidies- DELAY1 (Government subsidies, 1))/Government subsidies)
12. Rate of return on sale = IF THEN ELSE (Accumulated costs = 0, 0, (Accumulated revenues − Accumulated costs)/Accumulated costs) *∗* 100
13. Damage rate of goods = IF THEN ELSE (Transport time ≥ 2, 0.04 *∗* (2 − 0.6 *∗* Cold chain logistics technologies-0.4 *∗* Standardization), 0.02 *∗* (2 − 0.6 *∗* Cold chain logistics technologies-0.4 *∗* Standardization))
14. Quantities received by import enterprises = DELAY1 ((Amount of vegetables in transit I − Amount of damage in transmit for core enterprises) *∗* Qualified rate of quality inspection IV: Thai Customs inspection *∗* Qualified rate of quality inspection III: Yunnan Customs inspection, Transport time)
15. Vegetable quality = IF THEN ELSE (Transport time *∗* (2 − 0.5 *∗* Cold chain logistics technologies-0.5 *∗* Freshness grade of vegetables) ≥ 2, 0.5, 1)
16. Inventory of wholesalers = DELAY1 (Amount of vegetables in transit II − Amount of ex-warehouse in wholesalers, Transport time to markets)
17. Amount of vegetables in transit II = IF THEN ELSE (Inventory of import enterprises ≥ Market forecasting for vegetable sales, Market forecasting for vegetable sales, Inventory of import enterprises)
18. Average purchasing volume of primary wholesalers = RANDOM UNIFORM (430, 510, 0)
19. Market forecasting for vegetable sales = SMOOTH (Sales volume of vegetables, Time for quick response)
20. Quantities received by retailers = DELAY1 (Amount of vegetables in transit II − Amount of ex-warehouse in wholesalers, 1)
21. Amount of ex-warehouse in wholesalers = IF THEN ELSE (−Damage rate of transport + Predicted quantity demanded of retailers < Inventory of wholesalers, −Damage rate of transport + Predicted quantity demanded of retailers, Inventory of wholesalers)
22. Predicted quantity demanded of retailers = RANDOM UNIFORM (1360, 1410, 0)

The article "Impact of Closed Operation Strategies on Profit of Core Enterprise in Closed Supply Chain for Vegetables: A System Dynamics Approach" was published in 2022. Journal: Comput Intell Neurosci.

## 4. Simulation and Forecasting

### 4.1. Model Checking

As known to us, it is impossible for the model to achieve accurate prediction, but only forecast the future through reasonable assumptions based on the current situation. As long as the predicted changes are correct in the trend, the design of the model is considered to be feasible. The test of the system dynamics model mainly includes two aspects:

Firstly, consistency check of variable units: there are many variables in a system dynamics model, each of which represents a different meaning and a different unit. So, it is necessary to maintain the consistency of the variable unit in the model construction. Meanwhile, the check mode function in Vensim software has implications for user's model checking, which improves the efficiency of modeling. Aiming to maintain the consistency of units, the model in this study has been proofread repeatedly.

Secondly, validity and rationality test: as the interaction between the four subsystems, the hierarchical error transfer will be caused along the causal chain. Given the profits of vegetable supply chain change with the evolution, the predictions are likely to be different from their historical contribution. In previous studies, we usually compare the simulation results with the actual values of the same period to verify the validity and rationality of model. Generally, as long as the relative error between the simulated value and the actual one is less than 10%, the design of the model is reasonable [36, 38, 45]. In the field survey of 10 vegetable enterprises and interviews with 20 supply chain experts, we know that this standard is currently accepted by the industry. This method can reveal the changes of impact of simulation results on future profits for vegetable supply chain over time.

As mentioned earlier, *Capsicum frutescens* and broccoli have become the two most representative vegetables in the vegetable supply chain exported from Yunnan Province to Thailand, which are selected for simulation in this study. The simulated values in the model are tested in Tables 4 and 5.

From the comparison of simulated values and actual values of accumulated profits for broccoli and *Capsicum frutescens* in 180 days, we can see that the margins of error between the two ones are within 10%; that is to say, the hierarchical error of the model is within a controllable range; thus, the model shows good performance in simulation and prediction.

### 4.2. Simulation Results Analysis

The development trend of accumulated profits of closed supply chain for the two vegetables can be directly visualized through Vensim software, in which SM1 is the original scheme, the reality of accumulated profits for broccoli and *Capsicum frutescens* before the implementation of closed strategies. The trend of accumulated profits for broccoli and *Capsicum frutescens* under conventional development within 180 days is shown in Figures 10 and 11, respectively.

As can be seen from Figure 10, with the development of vegetables trade from Yunnan Province to Thailand, despite the impact of COVID-19, the accumulated profits of broccoli still show a steady rise with small fluctuations. In the first five days, it is way up from the lowest value of 1.138 million dollars to 5.064 million dollars and then rises steadily with micro moves. On the 180th day, the total accumulated profits reach 19.522 million dollars, compared with the actual profit of 1.138 million dollars on the initial day, the growth rate is 1615.47%, which accords with the reality that as one of the most typical Yunnan vegetables, and broccoli has become the rigid demand in Thailand markets. It follows that the accumulated profits of broccoli will keep growing with further supply chain operations.

The article "Impact of Closed Operation Strategies on Profit of Core Enterprise in Closed Supply Chain for Vegetables: A System Dynamics Approach" was published in 2022. Journal: Comput Intell Neurosci.

As can be seen from Figure 11, the accumulated profits of *Capsicum frutescens* also show a steady rise with small fluctuations under conventional development. Specifically, the lowest value is that of 480,414 dollars on the first day, while on the 180th day, the total accumulated profits reach 19.129 million dollars, and the growth rate is 3881.82%. This conforms to the reality that *Capsicum frutescens* from Yunnan Province is quite popular in Thai markets, because it fits the favor of taste for Thai people, and it is an essential ingredient to a daily necessity. Thus, it can be concluded that *Capsicum frutescens* has a potential profitability and its accumulated profit can efficiently keep rising with further supply chain operations.

As can be seen from Table 6, within 90 days, broccoli has increased 10.59 million dollars, while *Capsicum frutescens* has increased by 9.38 million dollars only; within 180 days, *Capsicum frutescens* has increased by 18.65 million dollars, while broccoli has increased 18.38 million dollars only. In the long term, the absolute distance will become larger. In addition, starting from 90 days to 180 days, *Capsicum frutescens* has increased 0.94 times, while broccoli has increased by 0.66 times only. Thus, it is apparent that *Capsicum frutescens* has more highly profitable in the long run.

### 4.3. Forecast and Analysis under Different Schemes

#### 4.3.1. Prediction Schemes

By improving and adjusting the current development pattern, this study forecasts the profit trend of both broccoli and *Capsicum frutescens* in 180 days after the implementation of closed strategies of vegetable supply chain, aiming to improve the profit of core enterprises in vegetable supply chain from Yunnan Province to Thailand. In order to make the adjusted schemes more targeted, according to the simulation results analysis before, the parameters of system dynamics model are adjusted mainly by enhancing the execution efficiency of the closed strategies. In this study, a total of 7 schemes are designed to improve the influence coefficients of SM2, SM3, and SM4. Further, SM5 is a combination of SM2 and SM3, SM6 is a combination of SM2 and SM4, SM7 is a combination of SM3 and SM4, and SM8 is a combination of SM2, SM3, and SM4. The changes in impact parameters of seven prediction schemes are shown in Table 7.

The article "Impact of Closed Operation Strategies on Profit of Core Enterprise in Closed Supply Chain for Vegetables: A System Dynamics Approach" was published in 2022. Journal: Comput Intell Neurosci.

#### 4.3.2. Profit Forecast under Different Schemes

*(1) Profit Forecast for Broccoli under Different Schemes*. The SD model is used to forecast the accumulated profits of 7 schemes, the results are shown in Figure 12. As can be seen from the results, SM8, namely simultaneously strengthening the implementation of information traceability system, certificate of market access, and multistage quality inspection, has the most significant impact on the accumulated profits of broccoli, and what makes the minimum impact on the accumulated profits of broccoli is SM1 (the original scheme). Meanwhile, the accumulated profits of SM8 are gradually exceeding those of SM1 from the 16th day. Up to the 180th day, compared with the original plan, the accumulated profits of SM8 have increased by 72.51%.

In the second and third places are SM6 and SM5. Compared with SM8, although the impacts of SM6 and SM5 are not as great as those of simultaneously increasing the influence coefficient of the three closed strategies on accumulated profits, they still have a significant impact on the growth rate of accumulated profits. The growth values of accumulated profits for SM6 keep a little higher than those of SM5 during the simulation period, and the accumulated profits in both cases exceed the original scheme SM1 on the 16th day and 29th day respectively. Up to the 180th day, compared with the original plan, the accumulated profits of SM6 and SM5 have increased by 47.71% and 43.71% respectively.

In the fourth and fifth places are SM7 and SM2. Although the early growth rates are close, from the 15th day onwards, the incremental difference of accumulated profits between SM7 and SM2 has widened, and the accumulated profits in both cases exceed the original scheme SM1 on the 8th day and 51th day respectively. By the 180th day, SM7 earns 2.21 million dollars more than SM2, and the accumulated profit ratio of the two schemes has increased by 35.01% and 23.75%, compared with the original plan.

Lastly, SM4 and SM3 play a certain role in the accumulated profits of broccoli whose influence on the growth rate is between SM2 and SM1. The value of accumulated profits for SM4 is higher than that of SM1 on the first day, and the accumulated profits of SM3 exceed SM1 on the 36th day. Up to the 180th day, compared with the original plan, the accumulated profits of SM4 and SM3 have increased by 17.86% and 13.62%, respectively.

According to the analysis above, the influence of the 8 schemes can be ranked as follows: SM8 > SM6 > SM5 > SM7 > SM2 > SM4 > SM3 > SM1. It shows that SM8 has the most obvious impact on the accumulated profits of broccoli. Therefore, the core enterprises should firstly consider simultaneously strengthening the enforcement of the three closed strategies when they implement the closed operation mode in the supply chain.

*(2) Profit Forecast for Capsicum Frutescens under Different Schemes.* Exactly like the simulation of the broccoli, the parameters are changed according to Table 7, and the accumulated profits of 7 schemes are predicted by SD model. The results are shown in Figure 13. As can be seen from the results, SM8, namely, simultaneously strengthening the implementation of information traceability system, certificate of market access, and multistage quality inspection, has the most significant impact on the accumulated profits of *Capsicum frutescens*, and it returns to profit since the 6th day. In addition, what makes the minimum impact on the accumulated profits of *Capsicum frutescens* is SM1 (the original scheme), and the accumulated profits of SM8 are gradually exceeding those of SM1 from the 21th day. Up to the 180th day, the accumulated profits of SM8 have increased by 174.16%, compared with the original plan.

The article "Impact of Closed Operation Strategies on Profit of Core Enterprise in Closed Supply Chain for Vegetables: A System Dynamics Approach" was published in 2022. Journal: Comput Intell Neurosci.

In the second place is SM6, which has a significant impact on the growth rate of accumulated profits. Similar to SM8, it turns into profits on the 6th day, and the accumulated profits of SM6 exceed SM1 on the 21th day. Till the 180th day, compared with the original plan, the accumulated profits of SM6 have increased by 135.52%.

In the third and fourth places are SM5 and SM7. As can be seen from Figure 13, the accumulated profits of SM5 in the early stage are less than that of SM7, and SM5 begins to make profits from the 9th day; however, SM7 has never been operating in the red during the simulation period. On the 121th day, the accumulated profits of SM5 exceeded those of SM7. Since then, the growth rates of both come close. Till the 180th day, the accumulated profits of SM5 and SM7 have increased by 83.08% and 75.21%, respectively, compared with the original plan.

In the fifth and sixth places are SM2 and SM4. The accumulated profits of SM2 in the early stage are less than those of SM4, and similarly to SM8 and SM6, SM2 returns to profit since the 6th day; however, SM4 has never been operating in the red during the simulation period. On the 90th day, the accumulated profits of SM2 exceeded those of SM4. Since then, the growth rates of both come close. Till the 180th day, the accumulated profits of SM2 and SM4 have increased by 57.17% and 47.14%, respectively, compared with the original plan.

The article "Impact of Closed Operation Strategies on Profit of Core Enterprise in Closed Supply Chain for Vegetables: A System Dynamics Approach" was published in 2022. Journal: Comput Intell Neurosci.

Lastly, SM3 plays a certain role in the accumulated profits of *Capsicum frutescens* whose influence on the growth rate is between SM4 and SM1. The accumulated profits of SM3 exceed SM1 on the 37th day. Up to the 180th day, compared with the original plan, the accumulated profits of SM3 have increased by 18.11%.

Thus, the influence of the 8 schemes can be ranked as follows: SM8 > SM6 > SM5 > SM7 > SM2 > SM4 > SM3 > SM1. It shows that, with the results of broccoli, SM8 has the most obvious impact on the accumulated profits of *Capsicum frutescens*, which inspires the core enterprises to firstly consider simultaneously strengthening the enforcement of the three closed strategies when implementing the closed operation mode in the supply chain.

### 4.4. Results Summary

For improving the profit of the closed supply chain for vegetables, the system dynamics model is applied in this section, and three closed strategies are designed into seven schemes. Then two typical vegetables, broccoli and *Capsicum frutescens*, exported from Yunnan Province to Thailand are chosen, and their accumulated profits under different schemes are simulated and forecasted, respectively. Through contrastive analysis, the development trends of the two vegetables come to the same conclusion, that is, simultaneously strengthening the three closed strategies enables the creation of the biggest economic benefit for the core enterprises. This finding provides a scientific and quantitative reference for decision-making of vegetable enterprises and government sectors.

## 5. Conclusion and Recommendation

As for the impact of closed operation strategies on profit of core enterprises in closed supply chain for vegetables, based on the data from expert consultation, questionnaire, and field survey, two of the most representative vegetables, broccoli and *Capsicum frutescens*, are selected for this study. The system dynamics model witnesses the completion of simulation in which the accumulated profits of each vegetable represent a general steady increasing trend during the simulation time. However, compared with the following seven schemes, the current development (original scheme) is not as ideal as expected in terms of profitability. In particular, the accumulated profits of broccoli and *Capsicum frutescens* in SM8 are about 1.7 times and 2.7 times than those of the original scheme, respectively. Such fact certifies that implementing closed strategies in supply chain members is a precondition to improve profits and competitiveness in the supply chain between Thailand and Yunnan Province. However, as the data shows, the Kunming-Bangkok Road inspires trade between Thailand and Yunnan Province in vegetables cargoes though the profits of core enterprises do not experience too much growth as expected. This is why this supply chain is not a real sense of “cash cow” but needs to be improved instead. In addition, as the profit forecast under different schemes implies, the profit of core enterprises in this supply chain is closely related with the closed strategies. The predication shows that if the three strategies are implemented simultaneously, the accumulated profits of broccoli and *Capsicum frutescens* could to be 1.7 times and 2.7 times, respectively, than those in conventional development in the off-season every year, which shows the optimistic view about the future potentials along this supply chain. Thus, if the closed strategies could be implemented effectively, the core enterprises in this supply chain would attract more profits than predicted; namely, the trade between Thailand and Yunnan Province would grow up with higher rate.

The article "Impact of Closed Operation Strategies on Profit of Core Enterprise in Closed Supply Chain for Vegetables: A System Dynamics Approach" was published in 2022. Journal: Comput Intell Neurosci.

However, this study still has some limitations. Firstly, since the method is applied from the downstream to upstream in the supply chain, the parameters in each subsystem of the SD model are macroscale aggregated. The subdivision can be improved, namely, considering more subdivided vegetable varieties and specific technologies of storage and transport. Secondly, due to the complexity of operations of vegetable supply chain and dispersion of relevant data, there are some assumptions and uncertainties when scenario design and prediction. For example, in all scenarios, we did not consider the situation of the impact of the COVID-19 on the member enterprises, and we chose a fixed and comparable level of supply and demand, although changes of these factors will affect the actual profits of whole supply chain, especially that of core enterprises. Thirdly, there is lack of a mathematical model constructed to analyze the closed effect of each strategy on quality and safety control for vegetables. Therefore, future research could be expanded and developed in the perspective of game theory.

## Figures and Tables

**Figure 1:** Top 10 vegetable varieties exported from Yunnan province to Thailand by quantity in 2020 (source: Ministry of Agriculture and Rural Affairs, China; Kunming Customs; field research).

**Figure 2:** Top 10 vegetable varieties exported from Yunnan province to Thailand by value of export in 2020 (source: Ministry of Agriculture and Rural Affairs, China; Kunming Customs; field research).

**Figure 3:** Framework of profit system for core enterprises.

**Figure 4:** Causal diagram of subsystem of inventory of processing enterprises.

**Figure 5:** Causal diagram of subsystem of qualified inventory in core enterprises.

The article "Impact of Closed Operation Strategies on Profit of Core Enterprise in Closed Supply Chain for Vegetables: A System Dynamics Approach" was published in 2022. Journal: Comput Intell Neurosci.

**Figure 6:** Causal diagram of subsystem of inventory of import enterprises.

**Figure 7:** Causal diagram of subsystem of inventory of wholesalers.

**Figure 8:** Causal diagram of profit system for core enterprises in vegetable supply chain.

**Figure 9:** Flow diagram of profit system for core enterprises in vegetable supply chain.

**Figure 10:** Trend of accumulated profits for broccoli under conventional development unit: U.S. dollar.

**Figure 11:** Trend of accumulated profits for *Capsicum frutescens* under conventional development unit: U.S. dollar.

**Figure 12:** Trend of accumulated profits for broccoli under different schemes unit: U.S. dollar.

**Figure 13:** Trend of accumulated profits for *Capsicum frutescens* under different schemes unit: U.S. dollar.

**Table 1:** Volumes and values of Yunnan's vegetables exported to Thailand from 2015 to 2020.

Year	Volume unit: ton	Value of exports unit: dollars (million)
2015	13,058	120
2016	15,926	110
2017	180,759	110
2018	175,505	100
2019	209,136	140
2020	241,045	192

Source: Kunming Customs.

**Table 2:** Comparisons between closed supply chain and other types of supply chain.

	Closed supply chain	Green supply chain	Agile supply chain	Lean supply chain	Virtual supply chain
Main target	Food safety and process control	Ecological environmental protection	Quick response to demand	Avoiding waste and cost optimization	Flexibility and organizational restructuring
Operation cost	Higher	Higher	Average	Low	Average
Flexibility	Average	Average	Stronger	Average	Stronger
Product safety	Stronger	Average	Average	Average	Average
The third party supervision	Necessary	Necessary	Needless	Needless	Needless
Stability	Stronger	Average	Average	Average	Low
Application	Agricultural products, proprietary, articles, dangerous goods, and drugs	Products of high hygienic standard and high export standards	Demand-pull and innovative products	Bulk cargo, process maturity	Demand-pull products

Source: it is categorized by author.

**Table 3:** Notation list.

Notation	Term
*P*_1_, *P*_2_	Price in the export (wholesaler) market
PR_1_, PR_2_	The profit rate of the core enterprise (wholesaler) as the inventory variable
CP_1_, CP_2_	Rate of change for profit of the core enterprise (wholesaler) as the flow variable
IP_1_, IP_2_	Indicated profit rate of the core enterprise (wholesaler) sensitive to demand/supply balance
EB_1_, EB_2_	Effective terms of demand/supply balance on profit rate of the core enterprise (wholesaler)
*B*_1_, *B*_2_	Demand/supply balance term in the export (wholesaler) market
*S*	Supply of the core enterprise
DS	The wholesaler's demand/supply in the export (wholesaler) market
*D*	Demand of retailers
Import	Import amount which is added to supply in the wholesale market
*s*_1_, *s*_2_	Sensitive of price to demand/supply balance in the export (wholesaler) market
*C*	Cost per unit of product

The article "Impact of Closed Operation Strategies on Profit of Core Enterprise in Closed Supply Chain for Vegetables: A System Dynamics Approach" was published in 2022. Journal: Comput Intell Neurosci.

**Table 4:** Comparison of simulated values and actual values of accumulated profits for broccoli unit: U.S. dollar.

Time (day)	1	30	60	90	120	150	180
Actual value	1.116M	6.908M	8.921M	13.33M	13.679M	16.085M	17.587M
Simulated value	1.138M	6.632M	9.456M	11.73M	14.637M	14.637M	19.522M
Relative error %	0.02	−0.04	0.06	−0.12	0.07	−0.09	0.11

**Table 5:** Comparison of simulated values and actual values of accumulated profits for *Capsicum frutescens* unit: U.S. dollar.

Time (day)	1	30	60	90	120	150	180
Actual value	500,431.3	4.557M	6.504M	11.206M	12.73M	16.496M	17.234M
Simulated value	480,414	4.374M	6.894M	9.861M	13.621M	15.011M	19.129M
Relative error %	−0.04	0.22	−0.03	−0.11	0.04	−0.12	0.1

**Table 6:** Comparison of accumulated profits between broccoli and *Capsicum frutescens* unit: U.S. dollar.

Variety	1 day	90 days (M)	180 days (M)	Growth rate (%)
Broccoli	1.138M	11.73	19.522	1615.47
*Capsicum frutescens*	480,414	9.861	19.129	3881.82

**Table 7:** Changes in impact parameter of prediction schemes.

Code	Scheme	Adjustable parameter	Changes	
			Original parameter (%)	Adjusted parameter (%)
SM 1	Conventional development	None	—	—
SM2	Strengthening the implementation of information traceability system	Implementation efficiency	0	50
SM 3	Strengthening the implementation of certificate of market access	Implementation efficiency	100	140
SM4	Strengthening the implementation of multistage quality inspection strengthening the implementation of multistage quality inspection	Qualified inspection rate I	97.1	98.5
		Qualified inspection rate II	90.5	95.5
		Qualified inspection rate III	98	100
		Qualified inspection rate IV	98	100
SM 5	SM2 information traceability system + SM4 multistage quality inspection	Implementation efficiency	0	50
		Qualified inspection rate I	97.1	98.5
		Qualified inspection rate II	90.5	95.5
		Qualified inspection rate III	98	100
		Qualified inspection rate IV	98	100
SM 6	SM2 information traceability system + SM3 certificate of market access	Implementation efficiency	0	50
		Implementation efficiency	100	140
SM7	SM3 certificate of market access + SM4 multistage quality inspection	Implementation efficiency	100	140
		Qualified inspection rate I	97.1	98.5
		Qualified inspection rate II	90.5	95.5
		Qualified inspection rate III	98	100
		Qualified inspection rate IV	98	100
SM8	SM2 information traceability system + SM3 certificate of market access + SM4 multistage quality inspection	Implementation efficiency	0	50
		Implementation efficiency	100	140
		Qualified inspection rate I	97.1	98.5
		Qualified inspection rate II	90.5	95.5
		Qualified inspection rate III	98	100
		Qualified inspection rate IV	98	100

Source: author's design from expert consultation and field survey.

The article "Impact of Closed Operation Strategies on Profit of Core Enterprise in Closed Supply Chain for Vegetables: A System Dynamics Approach" was published in 2022. Journal: Comput Intell Neurosci.

## Data Availability

The data used to support the findings of this study are available from the corresponding author upon request.

## References

[1] Han X. (2014). *Research on Agricultural Products Closed Supply Chain Operation Mode and Performance–--in the Example of Agricultural Leading Enterprises*.

[2] Liu B. L. (2017). Demonstration project of technology integration and industrialization of closed supply chain for green agricultural products. *Academic Report*.

[3] Yunnan Characteristic Agricultural Products Circulation Association (2020). Vegetable Industry Development in Yunnan Province in 2020. *Academic Report*.

[4] Kramol P., Villano R., Kristiansen P., Fleming E. (2015). Productivity differences between organic and other vegetable farming systems in northern Thailand. *Renewable Agriculture and Food Systems*.

[5] Kunming Customs Volumes and Values of Yunnan’s Vegetables Exported to Thailand from 2015 to 2020. http://kunming.customs.gov.cn.

[6] Yunnan Administration for Market Regulation Sampling Inspection Results for Vegetables in Yunnan Province in 2020. https://nync.yn.gov.cn.

[7] Jiao Z. L. (2011). Research of sealed supply chain strategy and basic features. *Logistics Sci-Tech*.

[8] Qiu Z. Q. (2010). Research on logistics network optimization of green agricultural products closed supply chain. *Doctoral dissertation of Southwest Jiaotong University, China*.

[9] Bastas A., Liyanage K. (2018). Sustainable supply chain quality management: a systematic review. *Journal of Cleaner Production*.

[10] Chandrasekaran N., Raghuram G. (2014). *“Agribusiness Supply Chain Management,” Taylor and Francis Group LLC*.

[11] Chopra S., Meindl P. (2016). *Supply Chain Management, Strategy, Planning, and Operations*.

[12] He Q. W., Liu L. (2019). Assessing performance of ‘agricultural supermarket docking’ supply chain under rural revitalization strategy. *Ecological Economy*.

[13] Ernan H., Elena K., Ma Z. W., Suresh S. (2018). Relationship-specific investment and hold-up problems in supply chains: theory and experiments. *Business Research*.

[14] Wongsprawmas R., Canavari M., Waisarayutt C., Waisarayutt C. (2015). Food safety assurance system for fresh produce production in Thailand: a review. *Quality Assurance and Safety of Crops & Foods*.

[15] Zhang Y. (2014). Research on vegetable circulation pattern of Tianjin based on closed supply chain management. *Journal of Tianjin Agricultural University*.

The article "Impact of Closed Operation Strategies on Profit of Core Enterprise in Closed Supply Chain for Vegetables: A System Dynamics Approach" was published in 2022. Journal: Comput Intell Neurosci.

[16] Naser A. A. (2007). Application of quality tools by the Saudi food industry. *The TQM Magazine*.

[17] Concepcion S., Montiflor M., Hualda L. T., Migalbin L. R., Digal L. R., Rasco E. T. (2004). Farmers’ misconceptions about quality and customers’ preferences: contributing inefficiencies to the vegetable supply chain in southern Mindanao. *ACIAR Proceedings*.

[18] Guo C. M. (2011). Development of quality and safety certification of agricultural products in China. *Bulletin of Biology*.

[19] Madurika H., Hemakumara G. (2015). GIS based analysis for suitability location finding in the residential development areas of greater matara region. *International Journal of Scientific & Technology Research*.

[20] Yang J. S. (2005). Analysis of cost structure of production input for pollution-free vegetables. *Issues in Agricultural Economy*.

[21] Lv B. (2010). Research on integration of vegetable supply chain. *Doctoral dissertation of Fujian Agricultural University, China*.

[22] Frank C., Zvi D., Jennifer K. R., David S. L. (2000). Quantifying the bullwhip effect in a simple supply chain: the impact of forecasting, lead times, and information. *Management Science*.

[23] Yang W. M. (2006). Research on structure optimization of Chinese vegetable supply chain. *Doctoral dissertation of Chinese Academy of Agricultural Sciences, China*.

[24] Liu W. H., Zhang C. Q. Research on the cost control method of the green agricultural product sealed supply chain based on the total process analysis.

[25] Sun X., Zhang C. (2008). Cost structure and benefit distribution of agricultural products circulation in China. A case study of vegetable circulation in Dalian. *Issues in Agricultural Economy*.

[26] Alam G. M. M., Khatun M. N. (2021). Impact of COVID-19 on vegetable supply chain and food security: empirical evidence from Bangladesh. *PLoS One*.

[27] Rakesh D. R., Bhaskar B. G., Vaibhav S. N., Balkrishna E. N. (2019). Improvement in the food losses in fruits and vegetable supply chain - a perspective of cold third-party logistics approach. *Operations Research Perspectives*.

[28] Wang L., Yang L., Yang W. M. (2016). Research on distribution optimization of vegetable green supply chain. *Food Research and Development*.

[29] Alfred S. Bayesian networks and food security: an introduction. Bayesian statistics and quality modelling in the agro-food production chain.

[30] Gong H. J., Zhang W. C. (2009). Establishment of management system model in closed supply chain for pollution-free vegetables. *Academic Periodical of Farm Products Processing*.

[31] Ahuja G. (2000). Collaboration networks, structural holes, and innovation: a longitudinal study. *Administrative Science Quarterly*.

The article "Impact of Closed Operation Strategies on Profit of Core Enterprise in Closed Supply Chain for Vegetables: A System Dynamics Approach" was published in 2022. Journal: Comput Intell Neurosci.

[32] Prahalad C. K., Hamel G. (1990). The core competence of the corporation. *Harvard Business Review*.

[33] Harland C. (1997). Supply chain operational performance roles. *Integrated Manufacturing Systems*.

[34] Bendiner J. (1998). Understanding supply chain optimization. *APICS-The Performance Advantage*.

[35] Ma S. H. (2000). The influences of core enterprise on the formation of strategic partnership in supply chain. *Industrial Engineering & Management*.

[36] Yang H., Li X., Ma L., Li Z. (2021). Using system dynamics to analyse key factors influencing China’s energy-related CO2 emissions and emission reduction scenarios. *Journal of Cleaner Production*.

[37] McCool S. F., Lime D. W. (2001). Tourism carrying capacity: tempting fantasy or useful reality?. *Journal of Sustainable Tourism*.

[38] Qiao W. G. (2019). Effectiveness analysis and improvement simulation of coal mine safety management under the background of big data. *Doctoral dissertation of China University of Mining and Technology, China*.

[39] Comparison Chart for Vensim Configurations. *Website of Vensim*.

[40] Yuan D., Zhang X. (2019). An overview of numerical methods for the first kind Fredholm integral equation. *SN Applied Sciences*.

[41] Lee J. W., Prenter P. M. (1978). An analysis of the numerical solution of Fredholm integral equations of the first kind. *Numerische Mathematik*.

[42] Maleknejad K., Saeedipoor E. (2017). An efficient method based on hybrid functions for Fredholm integral equation of the first kind with convergence analysis. *Applied Mathematics and Computation*.

[43] Zhang X. M., Yuan D. (2017). A niche ant colony algorithm for parameter identification of space fractional order diffusion equation. *IAENG International Journal of Applied Mathematics*.

[44] Sterman J. D. (2003). System dynamics: systems thinking and modeling for a complex world. *ESD Internal Symposium*.

[45] Tan Y. Y. (2010). Carrying capacity of marine resources, ecology and environment, and its application in bohai bay rim. *Doctoral dissertation of Ocean University of China, China*.

